# Development of Microneedle Patch Loaded with *Bacopa monnieri* Solid Lipid Nanoparticles for the Effective Management of Parkinson's Disease

**DOI:** 10.1155/2022/9150205

**Published:** 2022-08-10

**Authors:** Delna Joy, Jobin Jose, Shabana Bibi, Akshay Bandiwadekar, Gopika Gopan, Clara Mariana Gonçalves Lima, Talha Bin Emran, Fahad A. Alhumaydhi, Harsha Ashtekar, Sandeep D. S, Carlos Adam Conte-Junior

**Affiliations:** ^1^NITTE Deemed-to-be University, NGSM Institute of Pharmaceutical Sciences, Department of Pharmaceutics, Mangalore 575018, India; ^2^Yunnan Herbal Laboratory, College of Ecology and Environmental Sciences, Yunnan University, Kunming 650091, Yunnan, China; ^3^Department of Biosciences, Shifa Tameer-e-Millat University, Islamabad, Pakistan; ^4^Department of Food Science, Federal University of Lavras, Lavras, Minas Gerais, Brazil; ^5^Department of Pharmacy, BGC Trust University Bangladesh, Chittagong 4381, Bangladesh; ^6^Department of Pharmacy, Faculty of Allied Health Sciences, Daffodil International University, Dhaka 1207, Bangladesh; ^7^Department of Medical Laboratories, College of Applied Medical Sciences, Qassim University, Buraydah 52571, Saudi Arabia; ^8^NITTE Deemed-to-be University, NGSM Institute of Pharmaceutical Sciences, Department of Pharmacology, Mangalore 575018, India; ^9^Center for Food Analysis (NAL), Technological Development Support Laboratory (LADETEC), Federal University of Rio de Janeiro (UFRJ), Cidade Universitária, Rio de Janeiro 21941-598, Brazil

## Abstract

The demand for drug delivery systems (DDS) to treat Parkinson's disease (PD) is still high, and microneedle (MN) assisted transdermal DDS offers enormous potential. Herbal products for PD have been shown to have antioxidant effects in reducing dopaminergic neurons from degeneration. Here, we attempted to incorporate solid lipid nanoparticles (SLNs) of *Bacopa monnieri* into dissolvable microneedle arrays and evaluate its neuroprotective activity. The bloodless and painless microneedle arrays through the transdermal route deliver the drug across the blood-brain barrier at the desired concentration. The quality by design (QbD) approach was employed for optimizing the SLNs formulations. The mechanical strength, *in vitro* release studies, *ex-vivo* permeation investigation, skin irritation test, histopathological studies, biochemical studies, and behavioural tests SLNs loaded microneedle arrays were performed. The microneedle patches obtained were shown to be mechanically robust and were also found to be nonirritant with a decreased degree of bradykinesia, high motor coordination, and balance ability. Compared to systemic delivery systems, such an MN method can achieve a considerably lower effective dose and allow long-term home-based treatment.

## 1. Introduction

The nervous system is unparalleled in executing complex thought processes and behaviours [1]. The blood-brain barrier (BBB) is a significant barrier since it prevents the passage of molecules into the CNS [2]. The role of BBB serves as a crucial barrier between circulating blood and neural tissues. It protects the interior brain environment by keeping the interstitial fluid composition and CSF within very tight bounds, allowing neurons to conduct complex integrative activities [3, 4]. The tight connections between intercellular clefts and the restrictions in the paracellular pathway combine to generate well-regulated metabolic and transport barriers, which are essential in brain pathology. Neuroprotection is another crucial characteristic of the BBB [5–7]. Brain pathology, which can arise from Parkinson's disease, can result in an abnormality in the CNS's microvasculature, which is the BBB's essential characteristic. Parkinson's disease is a common neurodegenerative disease indicated by nonmotor and motor symptoms [8]. Parkinson's disease causes cognitive deterioration, sadness, anxiety, dysautonomia, and sleep difficulties. Anosmia (loss of smell) affects up to 90% of persons with Parkinson's disease, and it can develop years before symptoms appear [9]. Pharmacologically correcting striatal dopamine, though symptomatic, may be claimed to address Parkinson's disease biology [10].

Herbal/natural drugs, also known as phytochemicals, have many disadvantages in initial clinical testings, such as low stability, poor absorption, and so on. The limitations put forth by the traditional system of herbal medicines are rectified by the development of novel drug delivery systems [11]. Various novel systems such as liposomes, ethosomes, solid lipid nanoparticles, solid dispersions, matrix systems, microemulsions, and so on, have been used as a novel approach to delivering herbal drugs. The development of novel drug delivery systems for herbal drugs has many advantages in providing the drug at a predetermined rate. It also provides the drug at the appropriate destination of action in the body. This approach helps improve the bioavailability of herbal drugs and may reduce the chances of side effects caused by the drugs delivered. It also increases the efficacy of drugs and may enhance patient compliance also. The evolution of innovative drug delivery systems helped control pharmacokinetics, nonspecific toxicity, immunogenicity, biorecognition, and effectiveness of drugs. They are designed to obtain continuous drug delivery at a predictable rate for an extended period [12].

*Bacopa monnieri* (local name: Brahmi) is a medicinal plant (*Scrophulariaceae* family) and has been widely accepted as herbal medicine to treat various nervous disorders and improve memory and intellect. Multiple studies have presented the pharmacological status of *B. monnieri* extensively, and the behaviour has been attributed principally to the presence of distinctive saponins known as “bacosides” [13]. The emergence of nanotechnology has opened up new possibilities for overcoming the challenges with CNS targeting by traditional drug delivery methods [14]. It is beneficial to use a drug-loaded nanocarriers system to treat Parkinson's disease. Lipid-containing formulations such as solid lipid nanoparticles have been widely used to facilitate CNS targeting and resolve the factors obstructing therapeutic agent delivery through the BBB [15, 16].

Nanoparticles are colloidal vesicles, and natural/synthetic polymers are used to prepare nanoparticles; they are ideally suited to optimize the delivery of drugs and minimize toxicity. The essential parameters for the successful delivery of drugs through nanoparticles depend upon nanoparticles' ability to cross multiple anatomical barriers, release the drug in a sustained manner, and describe the stability of particles in the nanometer size [17]. Significant advancement has been made by applying different drug delivery systems such as solid lipid nanoparticles (SLNs) to treat diseases. SLNs provide controlled drug delivery by modifying dissolution rate, enhancing entrapped drug bioavailability, enhancing tissue distribution, altered pharmacokinetic parameters, and drug targeting via various application routes. The lipidic structure of SLNs, combined with their nano size, ensures appropriate affinity with biological membranes, resulting in increased transdermal absorption [18].

Transdermal drug administration is a viable alternative to hypodermic injection and a captivating option for oral drug delivery. Compared to oral drug delivery, transdermal delivery of the drugs has several advantages. This route is preferred mainly when the drugs have a significant first-pass effect that causes drugs to be metabolized prematurely. Transdermal drug delivery systems are noninvasive and self-administered [19, 20]. The fundamental problem with the transdermal method is that many drugs cannot quickly pass the stratum corneum layer for therapeutic effect. When a microneedle device delivers the therapeutic agent, drug molecules can cross the stratum corneum layer, allowing an adequate concentration of drug molecules to enter the skin. In developing a microneedle system, hundreds of microneedles are arranged in an array on a small patch to produce the desired therapeutic response. A microneedle system aims to build a micron-sized transport pathway with needles that are only a few microns in diameter. The drug is directly transported into the epidermis and then passes into the systemic circulation, showing therapeutic action until it gets to the target [21].

Micron-scale needles integrated on a transdermal patch have been proposed to combine hypodermic needles and transdermal patches to solve the unique constraints of both injections and patches [22]. The study aimed to develop, characterize, and evaluate the SLNs of *B. monnieri* loaded dissolvable microneedle patch as a potential neuroprotective agent for the effective management of Parkinson's disease. *B. monnieri* loaded SLNs were developed, and the optimized formulation was incorporated into microneedle developed using polydimethylsiloxane (PDMS) and polyvinyl alcohol. Finally, the entrapment efficiency, *ex vivo* skin permeability, histopathology studies, biochemical tests and ability to treat parkinsonian symptoms in the model animal, and skin irritation tests of the SLNs incorporated microneedles were determined.

## 2. Materials

Standard materials used for this study are *B. monnieri* purchased from Novel Nutrients Pvt. Ltd., Bengaluru, India. Polyvinyl alcohol was purchased from Sigma-Aldrich (USA). Glyceryl monostearate, Tween 80, chloroform, and methanol were purchased from Loba Chemie Pvt. Ltd., Mumbai, India. All the materials used in the study are noncytotoxic.

## 3. Methodology

### 3.1. Preparation of *Bacopa monnieri*-SLNs Using GMS

The required weighed quantity of *B. monnieri* and glyceryl monostearate were dispersed in the chloroform and methanol solution in 1:1 proportion. One millilitre of Tween 80 in distilled water was heated up to 75°C. The drug:lipid concentration was then introduced into the aqueous phase dropwise and kept underneath the magnetic stirrer. This dispersion was exposed to sonication at a magnitude of 50%. Sonication was performed for an optimized magnitude equivalent to 50 cycles with 5 pulses of time intervals. The nanodispersion produced was cooled and used for further studies [23].

### 3.2. Optimization of *Bacopa monnieri*-SLNs

To optimize the *B. monnieri*-SLNs, the formulation variables identified were drug: lipid ratio (W:W) and sonication time (min). The quadratic response surface design represented by the second-order polynomial model was used to investigate the effect of these independent variables on dependent variables, that is, particle size (nm), polydispersity index, and drug entrapment efficiency (%) by using Design Expert® software (version 11.0.3.0 64 bit, Stat-Ease, Inc., Minneapolis, MN, USA). Response surface methodology (RSM), a group of statistical and mathematical methods, helps carry out a systematic analysis of the formulations. Using response surface methodology, the technique allows optimizing the numerical parameters that can influence the response surface; existing relation between numerical parameters can be quantified at different levels with obtained response surfaces. The independent factors drug:lipid ratio (A, W:W) and sonication time (B, min) were selected at three different levels, low (−1), medium (0), and high (+1) for each factor resulting in a 3-level factorial randomized quadratic design with 10 experimental trials. The experimental design and the actual values of the independent variables are given in Table 1. The *p* > 0.05 significance level was chosen. The best formulation was chosen based on the software's recommendations, with the smallest particle size, PDI, and highest entrapment efficiency [24]. The optimized formula was subsequently turned into a microneedle patch that was characterized by a variety of factors.

### 3.3. Characterization of *Bacopa monnieri*-SLNs

#### 3.3.1. Mean Particle Size, Polydispersity Index (PDI), and Zeta Potential

With the help of a zeta sizer (Malvern Zeta Sizer, UK), the mean size of particles, particle size distribution, and zeta potential were measured. The measurements were performed in triplicate [25, 26].

#### 3.3.2. Entrapment Efficiency

The entrapment efficiency of SLNs was evaluated by using the centrifugation method. The SLNs dispersion-containing drug was centrifuged in a cold centrifuge for 90 minutes at 16,000 rpm. The supernatant was collected and filtered. The drug content was determined by measuring the absorbance spectrophotometrically at 269 nm after suitable dilution [27].

(1) $$\begin{array}{c} \text{Entrapment efficiency}=\frac{a-b}{\alpha }\times 100, \end{array}$$

where *a* = quantity of drug incorporated into the SLNs and *b* = unencapsulated amount of drug.

#### 3.3.3. *In Vitro* Release Studies

The in vitro drug release studies of SLNs were carried out by using Franz diffusion cell. This apparatus consists of two chambers separated by a cellophane membrane. The formulation was placed on the membrane via the top chamber. The lower portion of the chamber was filled with phosphate buffer pH 7.4 solution, and the temperature was maintained at 37 ± 0.5°C. At each time interval, 1 ml of sample was withdrawn, and sink condition was maintained by replacing with the equal volume of phosphate buffer pH 7.4 solution. The % drug release was determined by analyzing samples at 269 nm using a UV-visible spectrophotometer followed by suitable dilution with phosphate buffer pH 7.4 solution [27].

### 3.4. Fabrication of *Bacopa monnieri*-SLNs Loaded Dissolving Microneedles

The optimized formulation containing *B. monnieri*-SLNs was transferred into two-layered dissolving microneedles. The polyvinyl alcohol (PVA) was dispersed in the optimized *B. monnieri*-SLNs dispersion to make a 10% PVA solution. After that, the prepared drug-polymer mixture was poured into the PDMS mould. The mould was placed in a rotary shaker for 30 min to load the drug into the needles. The backing layer was prepared by pouring a 10% PVA solution in distilled water into the mould. The patch was allowed to dry overnight before being detached from the mould. The blank patch was prepared by casting the 10% PVA solution into the PDMS mould [28, 29].

### 3.5. Characterization of *Bacopa monnieri*-SLNs Loaded Dissolving Microneedles

#### 3.5.1. Fourier Transform Infrared Spectroscopy (FTIR)

FTIR spectra of pure drug, lipid, PVA, and the *B. monnieri-*SLNs loaded microneedle patch was carried out using FTIR (Bruker) for physicochemical characterization. The samples were placed in the sample holder, and the pressure arm was placed above the models to record the spectrum. The different samples were scanned with a spectral resolution of 4 cm^−1^ to acquire FTIR spectra in a wave number range of 4,000 to 600 cm^−1^. The spectra were analyzed for any incompatibility between *B. monnieri* and excipients used in the formulation [29].

#### 3.5.2. Mechanical Properties of Microneedle

To determine the mechanical properties of needles, fabricated MNs were inserted on parafilm layers (Parafilm M®, a mix of a hydrocarbon wax and a polyolefin), and the depth of insertion was observed under an optical microscope (Leica S9D Trinocular microscope). The size of pores formed on the first layer and the pores formed on the successive layers were used to assess the mechanical homogeneity of the MN [30].

#### 3.5.3. Scanning Electron Microscopy

The morphology of the fabricated microneedle patch was observed by scanning electron microscopy (SEM). Photo micrographic images were taken at random locations, at different magnifications, and analyzed with an SEM (SEM-EDAX: Jeol 6390LA/OXFORD XMX N, Tokyo, Japan) operated at a 20 kV acceleration voltage [30].

#### 3.5.4. *In vitro* Drug Release of Microneedle Arrays

The microneedle arrays inserted into a single layer of Parafilm M® were immersed into the donor compartment of the vertical Franz diffusion cell on one end; it was fixed on the receptor compartment. The 12 mL of pH 7.4 phosphate buffer medium was transferred to the receptor compartment and maintained at 37 ± 0.5°C. The 1 mL of the samples were collected at the fixed period from the receptor compartment; then, the exact amount was substituted with a fresh medium to retain sink conditions. The samples so obtained were analyzed through UV spectroscopy at 269 nm.

#### 3.5.5. *Ex vivo* Permeation Study

A two-compartment Franz diffusion cell was used for the *ex vivo* permeation studies. The donor compartment was covered with goatskin (procured from a local slaughterhouse and soaked previously). The drug-loaded MN patch was placed in the goat's skin and attached to the other end of the donor compartment. The reservoir compartment was filled with a dissolution medium and kept at 37 ± 50°C under stirring. One millilitre of the samples were withdrawn from the reservoir compartment at fixed time intervals for 8 h, and 1 ml of fresh phosphate buffer of pH 7.4 was replaced to maintain the sink conditions. The samples were analyzed by UV spectroscopy.

### 3.6. Determination of the Neuroprotective Activity of the *Bacopa monnieri-*SLNs Loaded Dissolving Microneedles

The male Wister albino rats (200–220g) were split into six groups, with six animals in each group. Rats were randomly allocated into four groups: (1) control group subcutaneous (sc. injections of saline for 5 days and then administered with blank microneedle patch once for another 7 days); (2) rotenone treatment group (sc. Injections of 2 mg/kg rotenone for 5 days and then administered with blank microneedle patch once for another 7 days); (3) rotenone and pure *B. monnieri* loaded microneedle patch treatment group (sc. 2 mg/kg rotenone injections for 5 days, then pure drug-loaded microneedle patch once for another 7 days); (4) rotenone and unloaded patch treatment group (sc. 2 mg/kg rotenone injections for 5 days, followed by unloaded patch administration for another 7 days); (5) rotenone and blank SLNs loaded patch treatment group (sc. 2 mg/kg rotenone injections for 5 days, followed by SLNs loaded patch administration for another 7 days); and (6) rotenone and *B. monnieri*-SLNs microneedle patch treatment group (sc. 2 mg/kg rotenone injections for 5 days, followed by *B. monnieri*-SLNs microneedle patch administration for another 7 days). Patches were given 24 h following the last rotenone injection, after which the rat's dorsal region was gently shaved and cleaned with warm water. Institutional Animal Ethics Committee approved the study, and the approval number is NGSMIPS/IAEC-June 2020/194.

#### 3.6.1. Behavioural Studies

*(1) Rotarod test.* The rotarod test is the behavioural method for evaluating a drug's effects on animal motor control and muscle coordination. It is significant for assessing chemical products that explain neurological depression in the model animal. Most of the joint assessment is on neuromuscular coordination and the behavioural changes in the model animal. This study allows for a quick and easy evaluation of a drug-loaded microneedle patch impacting neuromuscular coordination. The rats are evaluated here after being placed on the rod. Five rats could be tested simultaneously using the device, consisting of a five-lane spinning rod. Rats were placed on the rotating rod and measured fall time at 18 rpm [31, 32]. The fall time measurement will explain the central nervous system depression in rats.

*(2) Actophotometer.* The locomotor activity was measured using an actophotometer. The treatment for each animal was explicitly given and placed in an actophotometer, allowing them in the activity cage for 10 minutes. An activity count was taken when the beam of light landing on the photocell was cut off due to the animal's movement. The proportion of locomotor activity that increased or decreased was then calculated [33]. The central nervous system depression index was assessed on the basis of low proportion of locomotor activity.

#### 3.6.2. Biochemical Studies

*(1) Estimation of Reduced Glutathione (GSH).* One millilitre of 10% trichloroacetic acid was used to precipitate 1 ml of tissue homogenate to determine reduced glutathione levels. Four millilitre of phosphate solution and 0.5 ml 5,5-dithio-bis-(2-nitrobenzoic acid) (DTNB) reagent solution were mixed to a diluent of the supernatant, and absorbance was recorded at 412 nm. The glutathione is calculated as unit/mg protein.

*(2) Estimation of Catalase (CAT).* The supernatant was transferred to a tube and 0.045 mM hydrogen peroxide (H_2_O_2_) and 39 mM phosphate buffer. After mixing, the optimum density was recorded against a blank sample containing distilled water in the reaction mixture instead of homogenate. The CAT activity was measured by unit/mg of protein.

*(3) Estimation of Superoxide Dismutase (SOD).* The superoxide was measured using a spectrophotometric approach based on the xanthin assay, in which yellow nitroblue tetrazolium is turned to blue formazan EDTA, and then NBT is added to the reagent mixture, which is subsequently reacted with the sample. The absorbance of formazon chromophore was measured at 560 nm against the sample. Data were expressed as % inhibition.

#### 3.6.3. Histopathology Studies

To assess the extent of a substantia nigra (striatum) lesion. The mid-hemisphere of the brain was sectioned into longitudinal portions. The substantia nigra was established and fixed in 10% formalin for 24 h before being embedded in paraffin wax. Under a microscope, fixed substantia nigra tissue of 5 µm thickness will be stained with hematoxylin and eosin dye and examined for neuronal degeneration. In 10 microscopic fields, the area of neuronal degeneration was investigated. Under 10x magnification, histopathology images of different groups were observed [34, 35].

### 3.7. Skin Irritation Test

The albino rats were caged together and fed with laboratory food and water. To examine the irritation effects produced by the microneedle patches, the microneedle patch was placed on the back skin of a depilated rat, with the other side serving as a control. After the administration, the sites were observed for any signs of erythema and edema [36].

## 4. Results and Discussion

### 4.1. Preparation and Optimization of *Bacopa monnieri* Loaded SLNs

The SLNs of *B. monnieri* were formulated using different concentrations of glyceryl monostearate and other ingredients. Altogether 10 formulations of SLNs of *B. monnieri* were prepared and optimized using Design Expert® software.

### 4.2. Effect on Particle Size, Polydispersity Index, and Entrapment Efficiency

*Bacopa monnieri-*SLNs were prepared using different GMS concentrations and sonication time and characterized in particle size, polydispersity index, and zeta potential using Malvern Zetasizer. The quadratic model suggested 10 formulation batches varying the concentration of drug: lipid ratio and sonication time factors from the DOE approach. The results obtained for the dependent factors particle size, polydispersity index, and % entrapment efficiency for the experimental trials carried out using 3-level factorial design are shown in Table 2. The particle size of the 10 formulations ranged from 128 to 169; the polydispersity index ranged from 0.28 to 0.44, and % the entrapment efficiency was found to be in the range of 73.5–89. The RES (reticuloendothelial system) cells do not readily absorb nanoparticles and SLNs, mainly those particles with a size range of 120–200 nm. Therefore, the developed SLNs bypass the liver and the spleen filtration. The contour plot and the 3D surface plot for the response particle size are shown in Figures 1(a) and 1(b). From the figures, it was observed that as the concentration of drug-lipid increased, the particle size and PDI decreased to a certain level, further increase in the concentration of drug-lipid ratio caused an increase in particle size and PDI, and the effect of drug-lipid ratio was found to be less significant in comparison with the sonication time. As the sonication time was increased, the particle size and PDI was found to be reduced gradually; hence, the effect of sonication time on particle size and PDI was found to be more significant. The contour plot and the 3D surface plot for the response PDI are shown in Figures 2(a) and 2(b). The substantial mechanical shear-induced within the formulation system causes vesicles with smaller particle sizes to develop when a longer sonication duration is used. The high sonication time causes high cavitation intensities in the liquid phase, resulting in small size. On the other hand, lower sonication time promotes the formation of more giant vesicles due to the tendency of individual globules to merge. The contour plot and the 3D surface plot for the response % entrapment efficiency are shown in Figures 3(a) and 3(b). As the sonication time was increased, the % entrapment efficiency was found to increase constantly hence the effect of sonication time on entrapment efficiency (%) was found to be more significant. The drug entrapment efficiency increases as the lipid (GMS) content rises. Among all other formulations, the F9 formulation had the highest level of entrapment (89%). It is because a higher GMS concentration results in better encapsulation efficiency. The zeta potential value of the F9 formulation was −19.21 ± 0.89 also indicates good colloidal stability.

### 4.3. *In vitro* Drug Release Study

The dissolution rate of the drug determines the *in vitro* drug release profile. Out of all the formulations, the formulation F9 showed a maximum % *in vitro* drug release (79.21%), as shown in Figure 4. The F9 formulation had a better release due to increased lipid contents, contributing to the drug's quick diffusion. The inclusion of nanosized carriers may be responsible for the overall increase in dissolution rate. The improvement in drug solubility could be attributable to the SLNs' ability to change drug crystallinity to an amorphous state [37].

### 4.4. Fabrication of *Bacopa monnieri-*SLNs Loaded Dissolving Microneedles Patch

In terms of evaluation parameters, the formulation F9 was selected as the optimized formulation, and it was incorporated into microneedle arrays and evaluated for further studies. The microneedles were fabricated by the micromoulding method [29]. The prepared blank and drug-loaded patches are shown in Figure 5. The encapsulation of drugs into microneedle depends upon the density and concentration of the drug, the number of needle tips (225 tips), the base width of tips (0.2 mm), and tip height. The formulation density was found to be 0.1268 ± 0.33 mg/mm^3^. And the drug that can be localized in the needles was found to be 0.3904 ± 0.05 mg.

### 4.5. Characterization of *Bacopa monnieri*-SLNs Loaded Dissolving Microneedles

#### 4.5.1. Fourier Transform Infrared Spectroscopy (FTIR)

The drug-excipients compatibility was confirmed by observing the functional groups with peaks of standard ranges. The principle peaks identified for pure drug at 3,276 cm^−1^ are attributed to O–H stretching vibrations, 1,634 cm^−1^ to C=C stretching, and 661 cm^−1^ to C=C starching (group – alkene). The principle peaks identified for GMS at 2,955 cm^−1^ are attributed to O–H stretching (group – alcohol), at 1,737 cm^−1^ to C=O stretching (group-carboxylic acid) and at 1,270 cm^−1^ to CO stretching (group – ether). The principle peaks identified for PVA at 3,702 cm^−1^ attributed to O–H stretching vibrations (group – alcohol), at 1,762 cm^−1^ to C=O stretching (group – ester), at 1,428 cm^−1^ to S=O stretching (group – sulfonyl chloride), and at 3,082 cm^–1^ to C–H alkene (group – alkene). The principle peaks identified for the optimized formulation of microneedle patch at 3,335 cm^−1^ are attributed to O–H stretching (group – alcohol), at 1,719 cm^−1^ to C=O stretching (group – carboxylic acid), and at 664 cm^−1^ to C=C stretching (group – alkene). The principle peaks observed in FTIR spectra of *B. monnieri*, GMS, PVA, and the optimized formulation microneedle patch were found to be similar and within the acceptable range. It was confirmed that there was no incompatibility between excipients used in formulating the SLNs loaded microneedle patch. The FTIR spectral images of *B. monnieri*, GMS, PVA, and the optimized formulation microneedle patch are shown in Figures 6(a)–6(d), respectively.

#### 4.5.2. Mechanical Properties of Fabricated Microneedles

Microneedles were placed into a parafilm layers stack by an applicator for mechanical properties determination. Further individual layers were separated and inspected under an optical microscope to test the mechanical uniformity of microneedles (Figure 7). The pores formed were uniform in size, and pores on the second layer of parafilm showed consistent needle length. Furthermore, on the second sheet of parafilm, microneedles were pushed with more pressure, and the resulting pores were found to be identical in size. The hollow area suggested that only some microneedles can permeate the viscoelastic substance, whereas the solid area pointed to homogeneous needles [29]. The various properties such as the density of the needles, needle length, base dimensions, sharpness, material, and geometry all affected the penetrating properties of microneedles. Fig . 7 shows the optical microscopic photographs of a PDMS mold (Fig. 7(a)), a blank patch (Fig. 7(b)), and a Bacopa monnieri-loaded patch (Fig. 7(c)).

#### 4.5.3. Scanning Electron Microscopy

The scanning electron microscopy images showed that fabricated microneedles appeared as needle-like structures (Figures 8(a) and 8(b)). The SEM image in Figure 8(c) indicates that the microneedle had a sharp tip to insert microneedle into the skin. The developed microneedles had a square pyramid shape and a proper needle-to-needle distance. The SEM pictures further indicated that the dimensions did not alter after the drug was encapsulated.

#### 4.5.4. *In Vitro* Drug Release of Microneedle Arrays

The *in vitro* drug release profile was plotted, and the drug release was found to be 69.9% at the end of 8 h (Figure 9). And the obtained results were in line with the *in vitro* results of SLN. It had a burst release characteristic in the beginning and subsequently transitioned to a more steady release pattern.

The dissolving of microneedle tips in the dissolution medium caused the burst release.

According to Prabhu et al., once the dissolving is complete, holes in the parafilm allow the dissolution medium to permeate more slowly into the patch, allowing the drug to be released [37].

#### 4.5.5. *Ex Vivo* Permeation Study

The *ex vivo* drug permeation studies were carried out using excised goatskin using Franz diffusion cells, and from obtained results, the graph was plotted (Figure 10). The drug permeation was 57.45% within 8 h, which is in line with the *in vitro* results. The percentage release in the e*x vivo* permeation study was less than *in vitro* drug release study since the drug should permeate through the actual biological membranes. Microneedle penetration efficiency is determined by the skin's viscoelasticity, the drug's physicochemical properties, and microneedle geometries. The microneedles effectively rupture the stratum corneum, allowing the drug to diffuse through the microchannel and the dermis [37, 38].

### 4.6. Determination of the Neuroprotective Activity of the *Bacopa monnieri-*SLNs Loaded Dissolving Microneedles

#### 4.6.1. Behavioural Studies

Rotarod and actophotometer studies helped understand rotenone produced disturbance in motor coordination and locomotor behaviour. Actophotometer is widely used to assess locomotor activity in rodents. It is employed to test the effect of various pharmacological treatments and brain damage. The motor activity of disease control animals was reduced than control group animals that implicates the disease condition of animals [32]. The animals group treated with *B. monnieri* loaded SLNs incorporated microneedle patch showed improved motor coordination compared to the other groups (Figure 11).

Rotarod and actophotometer studies reveal that rotenone causes disturbance in motor coordination and locomotor behaviour. Compared to control and DC, the motor activity of animals is reduced, which implicates rats' disease condition. Cotreatment with *B. monnieri* and microneedles has elevated motor coordination than DC, blank patch, and SLNBP alone. In the behavioural test, drug SLNs loaded microneedle patch has shown better activity than pure drug. Thus, increase in motor coordination and balancing abilities may be due to the protective effect of the drug (*B. monnieri*) on dopaminergic neurons against rotenone-induced toxicity of Parkinson's disease. Therefore, the current study investigated the impact of the drug (*B. monnieri)* SLNs loaded MN patch on the locomotor deficit by actophotometer, and obtained results showed that the rotenone-induced group has demonstrated a reduction in the locomotor activity. In contrast, treatment with *B. monnieri-*SLNs loaded microneedle patch showed improved locomotor activity.

#### 4.6.2. Biochemical Studies

The mitochondrial redox environment is maintained by GSH, which acts as the primary antioxidant and detoxifying enzyme that inhibit or repair oxidative modifications. The rotenone-treated animals had significantly lower GSH levels in the brain than the control animal, as seen in Figure 12(a). Cotreatment of *B. monnieri* loaded microneedle patch and rotenone increased the level of GSH in the brain compared to the groups treated with rotenone alone, blank patch, and blank solid lipid nanoparticle loaded patch. The SLNPBM showed more significant results in preserving the level of GSH in the brain in rotenone‐induced toxicity when compared to pure drugs. In the brain, catalase activity was considerably reduced in the rotenone-treated group compared to the control group. Cotreatment with (*B. monnieri*) SLNs loaded microneedles patch and rotenone significantly enhanced the catalase activity compared to groups treated with rotenone alone, blank patch, and solid lipid nanoparticle loaded patch. In the SLNPBM group, the catalase activity was protected more in rotenone-induced damage in the brain when compared to *B. monnieri* alone (Figure 12(b)).

SOD activity was considerably lower in the rotenone-treated group than in the control group in the rat brain. Compared to rotenone-treated groups, cotreatment with (*B. monnieri*) SLNs loaded microneedles patch with rotenone dramatically increased SOD activity in the brain. The SOD activity in the brain was likely boosted more in the SLNPBM treated group than in the group treated with *B. monnieri* alone (Figure 12(c)).

In rats with rotenone-induced Parkinson's disease, delayed neuromuscular coordination declined locomotor activity, and loss of dopaminergic neurons was seen. Neurotransmitters are involved in various behavioural functions, including motor activity, cognition, and emotions. Following rotenone exposure, changes in the neurotransmitter dopamine levels have been found to cause histopathological changes in the brain related to motor functions in rats. In Parkinson's disease, pathological changes in the substantia nigra cause tremor, stiffness, and gait disruption with nonmotor symptoms. In the current investigation, rotenone treatment in animals reduced neuromuscular activity and decreased locomotor performance, indicating that rotenone compromised motor coordination. It has been reported that rotenone‐induced generation of reactive oxygen species production and mitochondrial damage are related to oxidative stress in the brain/SN/stratum neurons. An essential link between these two mechanisms can be the scavenging activity of CAT, SOD, and GSH against the accumulation of oxygen free radicals. Rotenone therapy decreased CAT, SOD, and GSH activities and enhanced oxidative stress in rats.

#### 4.6.3. Histopathology Studies

Brain histopathological studies were performed to assess the neuroprotective effect of *B. monnieri* directly. In histopathological findings, the section from the substantia nigra area of disease control animals' brains showed the intense degenerative neuronal cells having variable darkly stained nucleus (Figure 13(a), short arrow) with mild basophilic cytoplasm, neurofibrillary tangles (Figure 13(a), long arrow), focal reactive microgliosis (Figure 13(b), long arrow), and mild inflammation (Figure 13(b), short arrow). The moderate vacuoles in neuropils were seen in this section. In animals treated with *B. monnieri*, both normal (Figure 13(c), arrow) and degenerative neuronal cells having a dark nucleus with mild basophilic cytoplasm (Figure 13(d), arrow) were observed along with scant inflammation, and neuropils had focal vacuoles in this treatment group. In the test 1 treatment group, substantia nigra showed both normal (Figure 13(e), arrow), and degenerative neuronal cells having variable darkly stained nucleus (Figure 13(f), arrow) with mild basophilic cytoplasm, focal reactive microgliosis, and scant inflammation and neuropils were having mild vacuoles. In the test 2 treatment group, the section of substantia nigra showed both normal (Figure 13(g), arrow) and degenerative neuronal cells having variable darkly stained nucleus (Figure 13(h), arrow) with mild basophilic cytoplasm, focal reactive microgliosis, and moderate inflammation. The neuropils had mild vacuoles. In the test 3 treatment group, the section of substantia nigra showed both normal (Figure 13(i), arrow) and few degenerative neuronal cells having variable darkly stained nucleus (Figure 13(j), arrow) with mild basophilic cytoplasm and scant inflammation. Few congested blood vessels were also seen in this treatment group. Compared to a pure drug, the TDC:TNC ratio was significantly improved in the drug-loaded microneedle patch [33–35].

### 4.7. Skin Irritation Test

Wistar albino rats were used in the skin irritation test. After being treated with microneedles, there is no evidence of skin irritation or sensitivity as shown in Figure 14(a).  Figure 14(b) represents control rat skin, and Figure 14(c) shows the skin treated with a microneedle. As a result, the prepared microneedle patch was deemed safe as no irritation was found in animal skin.

## 5. Conclusion

The optimized SLNs dispersion was successfully incorporated into microneedle arrays for the transdermal delivery of *B. monnieri*. The microneedle patch of *B. monnieri-*SLNs was fabricated by micromuolding technique using polydimethylsiloxane (PDMS) moulds. The developed microneedle showed needle homogeneity, and the sharp pointed tip of the produced microneedles, as well as the square pyramid shape, aided skin penetration and retention during administration. The neuroprotective effect of *B. monnieri* was investigated on the rotenone-induced Parkinson's ‘disease rat *in vivo* and found that *B. monnieri-*SLNs loaded microneedle patch showed better neuroprotective activity when compared to the pure drug. The optimized formulation was tested for skin irritation on rat skin and showed no signs of irritation or sensitivity. The therapeutic efficacy of *B. monnieri* could be increased by developing it as a microneedle patch, boosting the drug's bioavailability via transdermal absorption.

## Figures and Tables

**Figure 1:** (a) Contour plot of particle size (nm) against drug: GMS ratio (w:w) and sonication time (min) and (b) 3D surface plot of particle size (nm) against drug: GMS ratio (w:w) and sonication time (min).

**Figure 2:** (a) Contour plot of polydispersity index against drug: GMS ratio (w:w) and sonication time (min) and (b) 3D surface plot of polydispersity index against drug: GMS ratio (w:w) and sonication time (min).

**Figure 3:** (a) Contour plot of entrapment efficiency (%) against drug: GMS ratio (w:w) and sonication time (min) and (b) 3D surface plot of entrapment efficiency (%) against drug: GMS ratio (w:w) and sonication time (min).

**Figure 4:** *In vitro* drug release profile of SLNs formulation.

**Figure 5:** (a) Blank patch and (b) *Bacopa monnieri-*SLNs loaded patch.

**Figure 6:** (a) FTIR spectra of *Bacopa monnieri*, (b) FTIR spectra of GMS, (c) FTIR spectra of Polyvinyl alcohol (PVA), and (d) FTIR spectra of microneedle patch.

**Figure 7:** (a) PDMS mould optical microscopic image, (b) blank patch optical microscopic image, and (c) *Bacopa monnieri* loaded microneedle image.

**Figure 8:** SEM images of (a) shape of drug-loaded microneedle patch, (b) needle to needle distance, and (c) the base diameter and height of microneedle.

**Figure 9:** *In vitro* drug release of the microneedle.

**Figure 10:** *Ex vivo* release data of microneedle patch.

**Figure 11:** Effect of treatment on locomotor activity and muscle strength. ^∗∗∗^ represents *P* < 0.05 versus the control group. Data represented as mean ± SEM (*N* = 6). C = control, DC = disease control, BM = pure *Bacopa monnieri*, BP = blank microneedle patch, SLNP = blank solid lipid nanoparticle loaded patch, and SLNPBM = *Bacopa monnieri* loaded solid lipid nanoparticle loaded patch.

**Figure 12:** (a) Effect of microneedle on cellular glutathione depletion and glutathione recovery in Wistar albino rats challenged with rotenone. Brain GSH levels were measured. The graph shows the protein present in unit/mg in brain homogenate, the degree of GSH depletion at DC, and the increase of GSH level in BM and SLNPM. Values given are mean ± SEM, with *n* (3). (b) Effect of microneedle on enzyme catalase depletion in Wistar albino rats challenged with rotenone. The graph shows the degree of reduced CAT at DC and increased CAT level in BM and SLNPM. Values given are mean ± SEM, with *n* (3). (c) Effect of microneedle on superoxide dismutase enzyme depletion in Wistar albino rats challenged with rotenone. The graph shows the degree of reduced SOD at DC and increase of SOD level in BM and SLNPBM. Values given are mean ± SEM, with *n* (3).

**Figure 13:** Histopathology studies: (a) disease control; (b) standard (pure drug patch); (c) test 1 (blank SLN patch); (d) test 2 (blank patch); (e) test 3 (drug+SLN patch). The ratio of TDC: total number of degenerative neuronal cells; TNC: total number of normal neuronal cells. TDC: TNC for the disease control group, 5.53:1; standard: 1:1.705; test 1: 1:2.21; test 2: 1.08:1; test 3: 1:4.5.

**Figure 14:** Control: (a) rat skin, (b) skin treated with a microneedle, and (c) skin after 24 h.

**Table 1:** Dependent and independent variables are taken in the optimization of formulations.

Factors	Levels, actual (coded)		
	−1 (Low)	0 (Medium)	+1 (High)
Independent variables			
A = drug: GMS ratio (W:W)	1:1	1:2	1:3
B = sonication time (min)	5	7.5	10
Dependent variables			
R1 = particle size (nm; R1)			
*R*2 = entrapment efficiency (%; R2)			
*R*3 = polydispersity index (R3)			

**Table 2:** DOE batches with results of particle size (nm), entrapment efficiency (%), and polydispersity index.

Formulation code	Factor 1 A: drug: lipid (w:w)	Factor 2 B: sonication time (min)	Response 1, particle size (nm)	Response 2, EE (%)	Response 3, PDI
F1	−1	−1	168	78.26	0.445
F2	0	−1	169	78.5	0.38
F3	1	−1	168	78.4	0.42
F4	−1	0	167	73.5	0.43
F5	0	0	146	81.4	0.37
F6	1	0	161	79.3	0.41
F7	−1	1	135	87.9	0.34
F8	0	1	139	85.3	0.36
F9	1	1	128	89	0.28

## Data Availability

The data used to support the findings of this study are included within the article.
